# Noninvasive Spectroscopic Detection of Blood Glucose and Analysis of Clinical Research Status

This article has been retracted.

**DOI:** 10.1155/2022/8325451

**Published:** 2022-02-07

**Authors:** Boqi Man

**Affiliations:** University College London, London, UK

## Abstract

Frequent measurement of blood glucose concentration in diabetic patients is an important means for diabetes control. Blood glucose monitoring with noninvasive detection technology can not only avoid the pain of patients and eliminate the harm of some biological materials for measuring glucose in vivo but also improve the frequency of detection, so as to control blood glucose concentration more closely. Traditional blood glucose detection methods are invasive and have some limitations. In this study, the significance of noninvasive blood glucose testing was analyzed and was pointed out that noninvasive blood glucose testing can monitor the blood glucose concentration of patients and relieve the pain of patients. Then, this study analyzed the spectral detection methods of noninvasive blood glucose, including conservation of energy metabolism, near infrared spectroscopy, and other spectral detection methods. Finally, this study made a comprehensive analysis of the domestic and international clinical application of noninvasive glucose spectrum monitoring and summarized the clinical application status of noninvasive glucose spectrum monitoring.

## 1. Introduction

Diabetes is a kind of disease caused by the deviation of blood sugar from normal value due to the disregulation of insulin secretion in human body, which is characterized by hyperglycemia [1]. At present, the main clinical treatment of diabetes is to adjust the amount of insulin injection through frequent monitoring of blood glucose concentration. Blood glucose tests are classified as invasive, minimally invasive, and noninvasive. In recent years, various countries are carrying out research on noninvasive blood glucose detection technology, and China has also invested a lot of manpower and material resources in this aspect. Compared with invasive and minimally invasive blood glucose concentration detection techniques, noninvasive spectroscopic detection of blood glucose can be used as a long-term detection method, which has the advantages of low cost, noninvasive, continuous real-time measurement, and so on [2]. Noninvasive blood glucose detection technologies are mainly divided into the following categories: near infrared spectroscopy, Raman light and other spectroscopies, human fluid extraction, impedance spectroscopy, conservation of energy metabolism, and so on; among them, the study found that there are many factors affecting blood glucose measurement by the energy conservation method, and the measurement accuracy is not high, so there is no market product based on the energy conservation method for blood glucose measurement [3]. In contrast, near infrared spectroscopy is a more mature technology for blood glucose measurement, which is also the focus of domestic and foreign scholars [4, 5]. Combined with the significance and method contents of noninvasive blood glucose spectrum detection, this study analyzed the status of noninvasive blood glucose spectrum detection and clinical research.

In this study, initially, the significance of noninvasive blood glucose testing was analyzed and was pointed out that noninvasive blood glucose testing can monitor the blood glucose concentration of patients and relieve the pain of patients. Then, this study analyzed the spectral detection methods of noninvasive blood glucose, including conservation of energy metabolism, near infrared spectroscopy, and other spectral detection methods. Finally, this study made a comprehensive analysis of the domestic and international clinical application of noninvasive glucose spectrum monitoring and summarized the clinical application status of noninvasive glucose spectrum monitoring.

The rest of the study is organized as follows. in Section 2, a detailed discussion is presented on the significance of noninvasive spectroscopic detection of blood glucose which is followed by conservation of energy metabolism in the next section. In Section 4, clinical application of noninvasive spectroscopic detection of blood glucose is presented along with various results and discussion. Finally, concluding remarks are given to provide a brief description of the overall activities which were carried out in this study.

## 2. Significance of Noninvasive Spectroscopic Detection of Blood Glucose

Whether invasive or minimally invasive, blood glucose measurement needs to collect blood or human interstitial fluid for measurement, which will cause physical discomfort to patients and may cause cross-infection, which greatly limits the possibility of popularization of these devices and fails to achieve continuous and real-time monitoring of every diabetic [6]. At this time, a convenient method for multiple measurements to achieve real-time monitoring of blood glucose is needed. Therefore, a series of studies on noninvasive blood glucose detection technology are carried out in this context. Noninvasive spectroscopic detection of blood glucose can achieve real-time and safe blood glucose concentration monitoring without the use of any consumables, reducing the cost of each measurement and reducing environmental pollution. At the same time, it is more easily accepted by people, so as to improve the frequency of blood glucose detection of patients and achieve more refined management of blood glucose concentration [7]. Noninvasive spectroscopic detection of blood glucose is a hotspot in current research, which has the following research significance:

1. Noninvasive spectroscopic detection of blood glucose can monitor the blood glucose concentration of patients in real time, enabling doctors to accurately and timely understand the condition of patients, so as to reduce the incidence of complications of diabetes patients.
2. Noninvasive spectroscopic detection of blood glucose can relieve patients' pain of frequent sampling during blood glucose testing, so as to improve patients' awareness of treatment and survival, reduce their mental burden, and enhance their ability to control the metabolic level [8].
3. Noninvasive spectroscopic detection of blood glucose can reduce medical costs, bring good economic benefits to the society, and avoid environmental pollution caused by blood collection. Most importantly, it can prevent the occurrence of blood infectious diseases.

## 3. Noninvasive Spectroscopic Detection of Blood Glucose

### 3.1. Conservation of Energy Metabolism

The conservation of the energy metabolism is used to measure blood glucose by the spectrometric method. The sensor used in the experiment consists of a light source and a photoelectric converter. When the finger is close to the light source, the incoming light source passes through the peripheral vascular system of the human body, and blood absorbs some of the light intensity, so the reflected light signal received by the photoelectric converter is attenuated [9]. The pulse changes periodically, which leads to the reflected light intensity that also changes periodically. The photoelectric converter converts the optical signal into electrical signal and amplifies and outputs it, so as to obtain the original data of photoelectric pulse wave. By establishing the mathematical model between pulse wave data and blood glucose, the blood glucose concentration can be calculated. A partial cut of the original pulse wave is shown in Figure 1:

The waveform obtained after filtering the original waveform and removing the baseline is shown in Figure 2:

According to the principle of spectrometric blood glucose measurement, the relationship between pulse wave and blood glucose concentration should be established. Principal component analysis (PCA) was used to reduce the dimension of the processed waveform data, and 6 characteristic parameters of the pulse wave were extracted, which are set to  *t*_1_, *t*_2_, *t*_3_, *t*_4_, *t*_5_, and *t*_6_, the mathematical function relationship of human blood glucose concentration is obtained:

(1) $$\begin{array}{c} BG={\text{f}}_{2}\left(t_{1},t_{2},t_{3},t_{4},t_{5},t_{6}\right). \end{array}$$

In the formula, *f*_2_ is a functional relationship, and  *t*_1_–*t*_6_ are the 6 feature parameters extracted after dimension reduction of pulse wave data. Combining the conservation of energy metabolism and the photoelectric volume pulse wave method to measure blood glucose, the functional relationship of blood glucose calculation can be obtained:

(2) $$\begin{array}{c} BG=f_{2}\left(T_{E},R_{H},T_{O},S_{O2},H_{R},t_{1},t_{2},t_{3},t_{4},t_{5},t_{6}\right). \end{array}$$

After establishing the above functional relationship, the blood glucose concentration can be calculated by using the corresponding algorithm model.

### 3.2. Near Infrared Spectroscopy

Near infrared spectroscopy is another technique for detecting the interaction between near-infrared light and tissue. Near infrared spectroscopy is commonly used to detect weak absorption in liquids and gases. In near-infrared laser pulses of 1 000–1 800 nm, tissues can be excited by the absorption of glucose molecules, resulting in fine local heating with light absorption [10]. The rise in temperature causes rapid thermal expansion, which creates a measurable ultrasonic pressure wave through a hydrophone or piezoelectric device in the tube or on the surface of the skin where it is located. The amplitude *P* of a pulse signal is associated with the absorption coefficient by the following formula:

(3) $$\begin{array}{c} P=\frac{K\left(\_aU\sqrt{v}\right)}{C_{\text{p}}}. \end{array}$$

In formulas (2) and (3), _*a* is the light absorption coefficient, *U* is the thermal expansion coefficient, *v* is the speed of sound, *C*_*p*_ is the intrinsic heat of the solution, and *K* is the proportionality constant associated with the macromolecules of the solute. With the increase of grape concentration, *C*_*p*_ in solution decreased, sound velocity increased. At the wavelength of glucose absorption, the change of PA signal is the result of the change of _*a*, *v*, and *C*_*p*_. When the total solute concentration changes, *v* and *C*_*p*_ values change. When PA is excited in the near infrared region, it detects the absorption caused by the doubling of the O − H and C − H band vibrations of glucose and other analyte, and the absorption is then converted into an acoustic pulse. The advantage of near infrared spectroscopy measurement over other near-infrared monitoring methods is its sensitivity, since the near infrared spectroscopy detector picks up all the generated signals in a single tissue and detects the generated signals at a longer wavelength range than the silicon or gallium arsenide monitor.

### 3.3. Other Spectral Detection Methods

In addition to conservation of energy metabolism and near infrared spectroscopy, other spectral detection methods include PA measurement, Raman measurement, optical rotation measurement, spatial decomposition diffuse reflection method, and so on [11]. In principle, noninvasive detection of human blood glucose concentration by the optical method is mainly based on the fact that changes in human blood glucose concentration will lead to changes in optical parameters of tissues. Therefore, the detection of changes in blood glucose concentration can be achieved by detecting optical parameters. The noninvasive spectral method of blood glucose detection obtains the information of blood glucose concentration by analyzing the changes in intensity, phase, polarization angle, and frequency after the light signal is applied to the detection site.

## 4. Clinical Application of Noninvasive Spectroscopic Detection of Blood Glucose

### 4.1. Clinical Application in China

In the research of noninvasive blood glucose detection using spectral technology, China started late and fell far behind the developed countries, but in recent years, some initial research has been gradually carried out. Inspired by the dual-wavelength noninvasive oximeter, Xi et al. [12] from Shanghai University of Traditional Chinese Medicine theoretically deduced the use of a limited number of near-infrared wavelengths to detect blood glucose concentration and established a mathematical model. Shen et al. [13] from Beijing Medical University used Fourier near infrared spectrophotometer to conduct a noninvasive test of blood glucose. Li et al. [14] from China Medical University have done some studies on glucose concentration in bovine blood by using near infrared spectroscopy. Chen [15], president of the Chinese Academy of Sciences, proposed a method of combining near-infrared spectroscopy with differential blood volume spectroscopy. Although this method has great difficulty in implementation, its breakthrough in principle is of great significance. Zhang et al. [16] combined with domestic and foreign research experience carried out some research work on the pressure between the light source probe and the measured part in noninvasive blood glucose detection and studied the application of the genetic algorithm and neural network algorithm in near-infrared noninvasive blood glucose detection.

Su et al. [17] from Tianjin University studied the relationship between the variation of skin scattering coefficient and blood glucose concentration and built an optical coherence imaging device. In order to reduce the interference of background noise and other components in human skin, Su et al. proposed a method of correlation coefficient calibration to solve this problem. By analyzing the correlation between the scattering coefficient and glucose concentration, the most relevant region can be obtained, and the prediction accuracy of the correction model of glucose concentration can be improved. Yu et al. [18] designed a dual-modulated polarization measurement system based on the principle of optical rotation to measure the concentration of glucose solution in simulated aqueous solution. The transmission spectra were collected by the NIR spectrometer through the front room device equipped with simulated chamber aqueous solution. The prediction errors of the two correction models were 18.9 mg/dL and 15.2 mg/dL, respectively. The experimental results show that the device can reduce the birefringence of the anterior chamber and achieve low precision measurement of glucose concentration in the aqueous fluid.

### 4.2. Clinical Application Abroad

The research of noninvasive blood glucose spectrum detection technology began in the middle of the last century. Due to its huge development prospect and application market, it has been a research hotspot in developed countries in recent decades. In the 1980s, Breithardt et al. [19] began experimenting with optical methods to measure the content of various components in the human body, but his research focused on the feasibility and patent applications of various optical methods. At the end of the last century, governments in many developed countries realized the potential of NIR noninvasive blood sugar detection and began to support research in this field [20]. Japan has invested 640 million yen in NIR noninvasive blood glucose testing and has formed a professional research institute with many well-known universities and enterprises. A large research group led by Professor Arnaud [21] used near-infrared spectroscopy to detect blood glucose information in human oral mucosa. The NIR noninvasive glucose research group has been established in the United States [22].

Henry's team studied the near-infrared diffuse reflectance spectrum of human oral mucosa in the 1111–1853 nm band, and the standard deviation of prediction of the glucose calibration model established by combining the single-individual OGTT experiment was 2.4 mmol/L [23]. Some scholars used a fiber optic probe to measure the diffuse reflection spectrum of fingers in the 800–1350 nm band. Combined with the data of a single individual, the SEP value of the calibration model was 2.0 mmol/L. Graf et al. [24] randomly collected the near infrared spectra of the arms of 7 patients with diabetes within the band of 1050–2450 nm within 35 days and selected the data of 3 patients to establish the calibration model. The obtained SEP value was 1.41 mmol/L. Tankasala and Linnes [25] studied the long-term stability of the calibration model in the NIR noninvasive blood glucose detection method. Sandia National Laboratories in the United States and The Haland Experiment Group in Mexico used the finger as the measurement site and the partial least squares method to establish the mathematical correction model. The root-mean-square error of the model is between 122 and 142 mg/dL [26].

## 5. Conclusion

In this study, initially, the significance of noninvasive blood glucose testing was analyzed and was pointed out that noninvasive blood glucose testing can monitor the blood glucose concentration of patients and relieve the pain of patients. To sum up, by using the noninvasive spectroscopic detection of the blood glucose method, patients can grasp their own blood glucose concentration anytime and anywhere, so that patients can accurately adjust the blood glucose concentration value, which is useful for treating diabetes and preventing diabetes complications and prolonging diabetes. The life expectancy of patients and the improvement of the quality of life of diabetic patients are of great significance. This study combines the significance of noninvasive spectroscopic detection of blood glucose, conducts in-depth research on the scientific issues and key technologies involved in noninvasive spectroscopic detection of blood glucose methods such as conservation of the energy metabolism and near infrared spectroscopy, and summarizes the clinical results of noninvasive blood glucose spectral detection application.

## Figures and Tables

**Figure 1:** A partial cut of the original pulse wave.

**Figure 2:** The waveform obtained after filtering the original waveform and removing the baseline.

## Data Availability

The data used to support the findings of this study are included within the article.

## References

[1] Ni L., Xue P., An C. (2021). Establishment of normal range for thromboelastography in healthy middle-aged and elderly people of weihai in China. *Journal of Healthcare Engineering*.

[2] Gurevich B. S., Dudnikov S. Y., Shapovalov V. V., Zagorskii I. G. (2019). Application of a spectroscopic method for noninvasive determination of glucose content in blood. *Russian Physics Journal*.

[3] Zhe W., Zhang B., Shi H., Zhao G., Wang N. (2020). Development of noninvasive blood glucose detection technology. *China Medical Equipment*.

[4] Xu Y., Deng C., Jiang X., Xu N., Wang Y.-M., Deng G. X. (2019). Application of OV-GA-BP neural network in blood glucose prediction. *Sensors and Microsystems*.

[5] Han G., Liu R., Xu K. (2018). Effective signal extraction based on differential floating reference measurement in nIR noninvasive blood glucose detection. *Spectroscopy and Spectral Analysis*.

[6] Barman I., Dingari N. C., Kang J. W., Horowitz G. L., Dasari R. R., Feld M. S. (2012). Raman spectroscopy-based sensitive and specific detection of glycated hemoglobin. *Analytical Chemistry*.

[7] Callery E. L., Morais C. L. M., Paraskevaidi M. (2019). New approach to investigate Common Variable Immunodeficiency patients using spectrochemical analysis of blood. *Scientific Reports*.

[8] Sim J. Y., Ahn C. G., Jeong E. J., Kim B. K. (2018). Microscopic photoacoustic spectroscopy for non-invasive glucose monitoring invulnerable to skin secretion products. *Scientific Reports*.

[9] Rogatkin D. A., Lapaeva L. G., Bychenkov O. A., Tereshchenko S. G., Shumskii V. I. (2013). Principal sources of errors in noninvasive medical spectrophotometry. part 2. Medicobiological factors of errors. *Measurement Techniques*.

[10] Jiasi W., Tao W., Zhao S., Zhao H. (2015). Feature extraction of photoacoustic signals for noninvasive blood glucose detection. *Electronic Design Engineering*.

[11] Lv P., Lu Z., He Q., Wang Q., Zhao H. (2019). Noninvasive detection of blood glucose in vivo based on photoacoustic spectroscopy. *Optics and Precision Engineering*.

[12] Mo X., Sun S., Yu X., Wang B. (1991). A mathematical model for continuous, noninvasive, quantitative detection of human blood glucose concentration. *Journal of Biomedical Engineering*.

[13] Shen T., Peng Q., Weng S., Zhou X., Wu J. (1996). Study on noninvasive measurement of blood glucose by Fourier time transform mid-infrared spectroscopy. *Spectroscopy and Spectral Analysis*.

[14] Li M., Sha X., Wang X. (2000). Noninvasive spectroscopic detection of blood glucose and clinical research status. *Biomedical Engineering Section*.

[15] Chen X. (1985). Using synchrotron radiation to measure the reflection and scattering of mirrors in vacuum ultraviolet and soft X-ray regions. *Acta Optics*.

[16] Zhang Y., Lv L., Xu K. (2005). Study on simulated samples for noninvasive blood glucose detection by near infrared spectroscopy. *Spectroscopy and Spectral Analysis*.

[17] Su Y., Meng Z., Yu H., Wang L., Liu T., Yao X. (2015). Study on delay time of human blood glucose balance by OCT noninvasive detection. *Laser Technology*.

[18] Yu Z., Qiu Q., Guo Y. (2013). Measurement of blood glucose concentration by optical rotation. *Laser Journal*.

[19] Breithardt G., Becker R., Seipel L., Abendroth R.-R., Ostermeyer J. (1981). Non-invasive detection of late potentials in man-a new marker for ventricular tachycardia. *European Heart Journal*.

[20] Arnold M. A. (1996). Non-invasive glucose monitoring. *Current Opinion in Biotechnology*.

[21] Arnaud C. (2006). Noninvasive glucose detection. *Chemical & Engineering News Archive*.

[22] Khan S., Rich P., Clifton A., Markus H. S. (2009). Noninvasive detection of vertebral artery stenosis. *Stroke*.

[23] Henry,Celia M. (2002). Noninvasive glucose detection.. *Chemical & Engineering News*.

[24] Graf I. M., Kim S., Wang B., Smalling R., Emelianov S. (2012). Noninvasive detection of intimal xanthoma using combined ultrasound, strain rate and photoacoustic imaging. *Ultrasonics*.

[25] Tankasala D., Linnes J. C. (2019). Noninvasive glucose detection in exhaled breath condensate. *Translational Research*.

[26] Kim A. H. M., Park B. H. S., Cho A. Y. (2014). Noninvasive deep Raman detection with 2D correlation analysis. *Journal of Molecular Structure*.

